This article has been retracted.

# Role of Phosphatidylinositol 3-Kinase and Its Catalytic Unit PIK3CA in Cervical Cancer: A Mini-Review

**DOI:** 10.1155/2022/6904769

**Published:** 2022-08-21

**Authors:** Guojuan Sun, Qiang Zhang, Yi Liu, Ping Xie

**Affiliations:** ^1^Ward Section of Home Overseas Doctors, Hospital of Chengdu University of Traditional Chinese Medicine, Chengdu 610072, China; ^2^Maternity Rehabilitation Center, Hospital of Chengdu University of Traditional Chinese Medicine, Chengdu 610072, China

## Abstract

In complicated disorders like cancer, signaling pathways form a tangled network. Targeting one gene may result in an unfavorable reaction from another off-target gene. Such entwined complexities may result in treatment resistance or failure in cancer patients. The PI3K/Akt/mTOR (phosphoinositol 3-kinase/protein kinase B/mammalian target of rapamycin) pathway is dysregulated in cervical cancer and is used as a biomarker for therapy. PI3K is a kinase that consists of a regulatory and catalytic domain and has phosphorylation capability. Class I components like the catalytic part (PIK3CA and PIK3CD) and regulatory part (like PIK3R1, PIK3R2, PIK3R3, and PIK3R5) are associated with oncogenesis and growth factors in cervical cancer. This review is aimed at discussing the involvement of the PI3K component of the PI3K/Akt/mTOR network in cervical cancer. Specifically, class I catalytic subunit PIK3CA has been identified as a pharmacological target, making it therapeutically significant. Apart from discussing the function of PI3K and PIK3CA in cervical cancer, we also discuss their inhibitors, which may be beneficial in treating cervical cancer.

## 1. Introduction

Cervical cancer affects the cervical tissues, i.e., the region connecting the vagina and uterus. According to the American Institute of Cancer Research, cervical cancer is the eighth most common cancer globally, with Swaziland showing the highest rate (Cervical Cancer Statistics |World Cancer Research Fund International (http://wcrf.org/). The estimated diagnoses of new cases by the American Cancer Society for 2021 in the USA are 14,480 and 4,290 fatalities (https://www.cancer.org/cancer/cervical-cancer/about/key-statistics.html). In the WHO European region, deaths from cervical cancer amount to ~28,000 women/year (WHO/Europe|sexual and reproductive health-cervical cancer).

Most types of cervical cancers are caused by HPV [1], with HPV16 and HPV18 primarily responsible for most of the cases [2]. Treatment is either surgery, radio, or chemotherapy [3]. Despite treatment, many patients die due to relapse or failure of therapy. It has been reported that the PI3K/Akt/mTOR pathway malfunctions in cervical cancer. Due to its significant role in cell growth and metabolism and others [4, 5], it is essential from a therapeutic point of view. It could also act as a biomarker for detecting cervical cancer [6, 7]. It is a class I component; PIK3CA is called a catalytic subunit [8] as it executes the function of PI3K and translates into p110*α* protein. PIK3CA mutations are found in 14–23% of cervical cancers [9]. We discuss the role of PI3K and PIK3CA in cervical cancer as follows.

## 2. PI3K and Its Catalytic Unit in Cervical Cancer

PI3K, a well-studied kinase, was identified over three decades ago, with initial research focusing on purification and cloning for oncoprotein association. In the second decade, the focus was on oncogenesis and activation/inhibition, while in the third decade, its direct contribution to cancer was confirmed through mutation-related studies [9]. It is delineated by its ability to phosphorylate the -OH group at the 3′ end of the inositol lipids. The substrate of class I PI3K is phosphatidylinositol 4,5 bisphosphate, which is phosphorylated to phosphatidylinositol 3,4,5 trisphosphate. This converted product transports pleckstrin homology (PH) domain-comprising proteins to the plasma membrane, such as PDK1 and Akt [10]. This is why Akt is reported in conjunction with the PI3K pathway in cervical cancer. In addition, mTOR has also been implicated in the pathway. It is also from the PI3K-related kinase family.

When PIK3CA was identified as an oncogene in a chicken virus in 1997, the direct involvement of PI3K in carcinogenesis was established. It demonstrated constitutive activation following fusing with the N-terminus's viral sequence, indicating its direct oncogenic potential [11]. According to the latest stats on the CBioPortal of Cancer Genetics (https://www.cbioportal.org/), PIK3CA expressed 35% of cervical cancer, 38% in cervical cancer squamous cell carcinoma, and 39% in cervical adenocarcinoma.

## 3. PIK3CA Mutations and Cervical Cancer

Currently, cBioPortal shows 1,625 occurrences of mutations in this gene in various cancers. In cervical squamous cell carcinoma, 77 missense mutations are listed, with 70 listed as driver and 7 having unknown significance. Twenty-five mutations show amino acid change, with varied copy numbers (Table 1).

Gene PIK3CA is augmented in cervical cancer, and somatic mutations in it have been linked with tumor formation in several cancers, including cervical cancer [3]. Increased copy number is also connected with a higher chance of cervical cancer [12]. Mutations in PIK3CA activate the PI3K/AKT/mTOR pathway. The discovery of somatic (tumor-specific) mutations has put PI3K into the limelight as vital to cancer. In addition, this discovery has revealed the potential of PI3K as a potential drug target. The highest number of missense and gain mutations was observed for squamous cell carcinoma (Figure 1). This has been reported by Xiang et al. [13] for the Chinese population as well, that a higher number of PIK3CA mutations exist in the squamous cell carcinomas (15.3%) compared to nonsquamous cell tumors (7.3%). Japanese population showed 5.6% somatic mutations in squamous cell carcinoma and a similar number in cervical adenocarcinoma. However, a higher amplification of this gene was observed in adenosquamous carcinomas (20.7%) than in cervical squamous cell carcinomas (1.4%) [14]. In a European cohort, 40% dominant oncogenic alterations were seen in PIK3CA [15], and in a North American cohort, PIK3CA mutation frequency was 23% in tumors [16]. In a US cohort, PIK3CA was most mutated in tumors of the cervix, but no difference was observed in squamous cells of adenocarcinoma [17].

## 4. PIK3CA Mutations concerning Cervical Cancer Prognosis

Several inhibitors of PIK3CA (Table 2) are being tried in patients. PI3K inhibitor buparlisib (BKM120) has been tested in cervical carcinomas at stages I, II, and III [9]. Since the PI3K pathway is involved in cisplatin resistance and radioresistance [18], we also looked for mutations in its catalytic unit that could alter therapeutic outcomes. It was reported that French patients with PIK3CA mutation hoarding tumors did not effectively respond to the cetuximab treatment [19].

Arjumand et al. [20] found that E545K-mutant PIK3CA cell lines are resistant to cisplatin and/or radiation treatment compared to the wild type. Inference from the Cancer Genome Atlas data also showed that an increase in PIK3CA tumor mutation might cause immunotherapy sensitivity in the squamous cervical carcinoma [8]. Recently, Li et al. inferred that mutant PIK3CA, in conjunction with fascin actin-bundling protein 1 (FSCN1), shows radioresistance [21]. PIK3CA mutations have been linked with overall survival in stage IB (tumor size 5 mm depth, 3 cm width) and II (that extends beyond the cervix) carcinoma [22]. Lachkar et al. have reported that better cancer-specific survival is observed in patients with wild-type PIK3CA while poor in mutated PIK3CA-bearing patients. Subsequent survival analyses revealed that PIK3CA mutation was a significant prognostic factor for poor overall survival (OS) [18, 22].

A study conducted on North American cervical cancer patients harboring PIK3CA mutations shows that these patients had an amplified death risk. However, copy number variation did not impact survival outcomes [16]. Biopsy results of Hong Kong Chinese patients have revealed that PIK3CA mutations are allied with tumor size and patient survival [23]. In the US cohort, it was seen that PIK3CA mutations were concomitant to a shorter survival, i.e., ~67 months, compared to ~90 months in patients that did not have any PIK3CA mutation [17]. Oaks et al. demonstrated in another US patient cohort that PIK3CA mutations were not linked with disease-free survival, but survival outcomes were impacted if the tumor comes from older patients [24]. Pergialiotis et al. [25] conducted a meta-analysis on mutations of PIK3CA and their connection with the survival of cervical cancer patients. Cumulated data of 12 studies with more than 2000 patients showed an inconclusive result. The bulk of the studies showed an association of deleteriousness with PIK3CA mutations in squamous cell cervical carcinoma.

## 5. PIK3CA Mutation Rate regarding Cervical Cancer in Different Populations

Liquid biopsy of PIK3CA mutations in the cell-free DNA of Hong Kong Chinese women was allied with the size of the tumor and survival outcomes. Around 22% of patients depicted E545K mutation in the PIK3CA gene [23]. In another study on the Chinese population, 13.6% of women showed this gene alteration in cervical cancer [13], while this number was reduced to ~8% nonsynonymous mutations in Swedish women [26]. In the US, around 11% of PIK3CA mutations were found in cervical adenocarcinoma and 5% in cervix squamous cell carcinoma [27]. A study on the Philippine population revealed that PIK3CA gene mutations were around 11% in cervical cancer patients. In comparison, the group negative for HPV had a frequency of 28.57% alterations in this gene while the HPV-positive group had a 4.76% mutation frequency [28]. In the Indonesian people, PIK3CA was mutated in 24% of patients [29]. In South Indian women, no alteration was found in this gene in cervical cancer [30]. In a study by Femi, 25.4% of samples from the White population, 21% from Asians, 31% from Black/African-Americans, and 62.5% from American Indians or Native Alaskans carried a PIK3CA mutation. In comparison, amplified gene presence was 18.9% for White, 21% for Asians, 28% for Black/African-Americans, and 12.5% for American Indians or Native Alaskans [31]. This number was 31% for squamous cell carcinomas in Latin Americans and 24% for adeno/adenosquamous carcinomas [32].

## 6. PIK3CA MicroRNA Profile in Cervical Cancer

Nair et al. [33] used an NGS and microarray assay to find cervical cancer miRNAs linked with several pathways and genes. In cervical cancer, they discovered that four miRNAs were elevated and seven were downregulated in the PIK3 pathway, specifically miR-429 and miR-363 influenced the PIK3CA gene via the PI3K/AKT route, and miR-5572 affected the PIK3CA gene via the mTOR pathway. TargetScan (http://www.targetscan.org/) [34] of the PIK3CA gene showed three conserved miRNAs in vertebrates. These were searched for cervical cancer in the literature, and we found that miR-152 was upregulated in cervical cancer. It could act helpful in diagnosis and linked with treatment outcomes [35]. Recently, Chen et al. [36] reported that miR-148a suppressed cervical cancer cell proliferation, but they linked it with genes other than PIK3CA. Since we know by data mining from the TargetScan database that this miRNA is linked with PIK3CA, it is most likely that it impacts cervical cancer in alliance with this gene.

Liangjun et al. [37] reported that miR-148a possibly reduces chemoresistance of cervical cancer HeLa cells to cisplatin. miR-148b also acts as a tumor suppressor and reduces cell proliferation and invasion capabilities, but Mou et al. described this concerning caspase activity [38]. However, again we could link it with PIK3CA function in cervical cancer based on a prediction, but the experimental role remains yet to be elucidated. These were the top three miRNAs predicted by TargetScan to be conserved in vertebrates. Details of other miRNAs that could act on PI3KCA were conserved in mammals and indicated by this database were matched with cervical cancer via the miRCancer database (http://mircancer.ecu.edu/). miRNAs exhibiting experimental evidence have been shown in tabulated form below (Table 3).

### 6.1. Limitations of the Present Study

Little is known regarding the impact of different PI3K isoforms on TME function in CLL. In contrast, numerous clinical trials studying novel PI3K inhibitors, dual PI3K*δ* and -*γ* inhibitors, and pan-Class IA inhibitors have been launched. Phosphatidylinositol 3-kinases (PI3Ks) are promising targets for potential anticancer drugs. Several classes of potent and selective small-molecule PI3K inhibitors have been developed in recent years, with at least fifteen compounds progressing to clinical trials as new anticancer medicines. Among these, idelalisib appears to be effective as a single agent and in conjunction with standard therapy in various nonlymphoma Hodgkin's subtypes. Clinical trials in phase III are currently recruiting volunteers.

## 7. Conclusion

Cervical cancer is a particularly severe kind of female cancer that claims thousands of lives each year worldwide. It is regulated by the PI3K network of components, with the catalytic unit of this kinase playing a critical role in this disease. A considerable fraction of patients show mutations in this region. We have listed the mutations and their types that could impact the PIK3CA unit and cervical cancer. Most of the patients harboring these mutations show resistance to chemo and radiotherapy. Furthermore, if these mutations are present in their tumors, many have a shorter survival period. A further element, however, has been linked: old age. However, the relationship between ethnicity and patients' genetic makeup is still being investigated, necessitating a genome-wide association study. In addition, therapeutic outcomes in cervical cancer patients with noncoding elements like microRNAs and lncRNA also remain to be studied.

### 7.1. Future Directions

Future trials combining innovative small-molecule inhibitors against different signaling pathways and these inhibitors with biological and pharmacological agents may improve their clinical efficacy even more. As a result, detailed analyses of the TME in these trials are required to explain the role of PI3K class I isoforms in the function of different cell types and to ensure that PI3K inhibitors may be used as a highly active, safe, and tolerated therapy option in cervical cancers.

## Figures and Tables

**Figure 1:** Type of PIK3CA mutations in various cancers of the cervix. Somatic mutations observed are shown. Green dots represent each case of the indicated mutation, and purple and black dots represent truncating alterations.

**Table 1:** PIK3CA missense mutations show the amino acid change in the cervical squamous cell carcinoma (*n* = 25).

Mutation	Copy number	Position
E542K	Gain/diploid/Amp	178936082
E545K	Gain/diploid/Amp	178936091
Q546R	Gain	178936095
E545Q	Diploid	178936091
H1047R	Diploid	178952085
R88Q	Diploid	178916876
R93W	Gain	178916890
R38H	Diploid	178916726
E453K	Gain	178928079
C420R	Gain	178927980
G106V	Gain	178916930
H1047Q	Diploid	178952086
C90R	Gain	178916881
V344G	Diploid	178921549
R115P	Diploid	178916957
E81K	Gain	178916854
E726K	Amp/Gain	178938934
L339I	Diploid	178921533
L866F	Diploid	178947162
R693H	Diploid	178938836
Q75E	Diploid	178916836
A339T	Gain	178927432
Y432C	Diploid	178928017
D589N	Diploid	178937377
H1047L	Diploid	178952085

**Table 2:** Inhibitors of PIK3CA approved or being tested against cervical cancer.

Drug	Trial status	Location
TQ-B3525	Recruiting	China
Radiation (volumetric arc radiotherapy, interstitial brachytherapy), cisplatin, and gemcitabine	Recruiting	Azerbaijan
AZD5363	Active but not recruiting	UK, USA, Spain, Netherlands, Singapore, Japan, Denmark, France, Canada
Copanlisib and taselisib	Recruiting	USA, Puerto Rico
RMC-5552	Active and recruiting at several centres	USA

Source URL: https://clinicaltrials.gov/ct2/results?cond=Cervical+Cancer&term=PIK3CA.

**Table 3:** PIK3CA miRNAs mined from the TargetScan database with a putative role in cervical cancer.

miRNA	Impact	Reference
miR-320	Downregulated and suppresses migration/invasion of cells	[39, 40]
miR-134	Downregulated and acts in alliance with lncRNA NCK1-AS1	[41]
miR-758	Downregulated and inhibits proliferation/metastasis of cells	[42, 43]
miR-186	Downregulated and promotes malignancy and promotes cancer by acting in alliance with lncRNA ANRIL	[44, 45]
miR-374	Downregulated and reduces proliferation	[46–48]
miR-340	Downregulated and suppresses metastasis	[49]

## Data Availability

No data is associated with this article.
